# Application of Artificial Intelligence Combined with 5G Technology in the Reform of English Teaching in Universities

**DOI:** 10.1155/2022/5203066

**Published:** 2022-05-25

**Authors:** Can Liu, Xia Sun

**Affiliations:** ^1^School of International Education, Guizhou Normal University, Guiyang 550001, Guizhou, China; ^2^Department of Foreign Language, Hefei Normal University, Hefei, Anhui 230061, China

## Abstract

The language assistance and learning sectors have currently undergone restructuring in the period of fifth-generation (5G) communication and artificial intelligence, influenced by technologies, cloud services, learning techniques, speaker identification, language processing, virtual environments, expanded actuality, and blended actuality. This study proposes a routing protocol of modernized energy-optimized low-energy adaptive clustering hierarchical protocol (M-LEACH) using artificial intelligence and 5G Internet technologies for online English teaching. A dataset of 6,600,000 items, containing 3,250,000 favorable and unfavorable texts in English, is employed. The dataset is preprocessed using normalization to eliminate the impulse noises. Discriminant features are extracted using a variational autoencoder (VAE), and a random forest (RF) classifier is used to classify the features with accurate performance. The performance of the protocol is measured in terms of transmission rate, alive nodes, energy consumption, and a number of transmitted packets. Results show that the proposed M-Leach protocol provides a high transmission rate, maximum transmitted packets, more alive nodes, and minimum energy consumption as compared to other protocols. The proposed protocol will transform online English teaching from closed to open, and passive to active learning, dramatically changing the time and space scenarios, as well as the supply levels of English education.

## 1. Introduction

The development of artificial intelligence and 5G in language recognition and natural language processing has also exerted a great influence on English language teaching. The technological products of artificial intelligence and 5G are bound to bring about changes in the college English teaching model. With the improvement of the online teaching model, teachers will have a difficult time collecting, analyzing, and processing bid data as online education and their efficiency will suffer [1]. Artificial intelligence and 5G, on the other hand, can address these challenges in a systematic and time-efficient manner. As a result, technology serves as the foundation for exploring changes in teaching models. The capacity to grasp and successfully apply new technologies like artificial intelligence can effectively overcome the problem of a single college English teaching model [2].

With the constant restoring the ability, the rapid growth of research and methodology, and the extensive utilization of the web and Internet in the study, academic institutions are facing greater challenges the teaching to be modernized, making it necessary to use PCs to handle digital learning. Training has been transformed by the growth of the Internet. The use of the Internet to teach has grown in popularity [3]. Because of the expansion of cloud computing, competent students may now easily use visual net innovation to create an optimum learning environment. In addition to being an auxiliary tool, the Internet serves as a primary source of intelligence, an educational medium, and a communication medium. Employing technology to carry out web education is a key mechanism for learners and lecturers to adjust to the demands of the advanced educational arrangement and promote logical and regulated instructions. [4].

The widespread availability of mobile Internet has created an English teaching environment for students, while big data networks geared to smart education and artificial intelligence (AI) have assisted in the creation of new English teaching theories and methodologies. Under the influence of blended learning, web-based classes, mini-classes, and other new learning techniques, English teachers must improve instructional strategies, begin reversing the relationship with students, and shift educators from rulers to advisors, with students becoming the most important factor influencing the success of English instruction. [5].

This study introduces a routing protocol called modernized energy-optimized LEACH protocol (M-LEACH) using artificial intelligence (AI) and 5G net technologies. A dataset of 6,600,000 items, containing 3,250,000 favorable and unfavorable texts in English, was employed. The dataset is preprocessed using normalization to eliminate the impulse noises. After that, the features are extracted by the VAE, and an RF classifier is utilized for the classification of these features with accurate performance. Finally, the performances are examined, and the result is compared with other existing methods.

The rest of the manuscript is organized as follows: Section 2 provides an overview of the existing works.  Section 3 illustrates the proposed method. The results are presented in Section 4, and the conclusion is given in Section 5.

## 2. Related Works

The continuous development and progress in information technology have also impacted English education. Individual variations among students are not taken into account in the traditional uniform English instruction model. To advance to a new stage in English education, the method of English education must break through and innovate, employing information technology to encourage student's enthusiasm for learning. In a recent study, Sun et al. [6] summarized the processes and measurements for incorporating “5G” innovation into Internet verbal education, as well as a qualitative research design for investigating the modern web audio lesson plan, describing the benefits, and suggesting remedies to the drawbacks. Hong et al. [7] used the web and AI techniques to examine a clear, convenient, and high-performing academic instructional data system that can address the needs of educators and students. Qian et al. [8] proposed a new multipurpose English speech recognition system. They collected audio English data and defined three key functions in this corpus, namely, three separate categorization functions for evaluating participants' physical and/or mental health, namely, sleep quality, fatigue, and stress. The standards are created using both classic machine learning methodologies and cutting-edge deep learning models. In [9], the authors developed an intelligence-aided scheme to expand the scale and scope of today's digital tech's implementation in university English cultural learning, as well as to manipulate the vast applicability of advanced technologies in university English cultural education, thus setting up a new path and opportunity for academy English cultural teaching. Lei [10] has presented an optimized technique for overcoming the challenges and adversity of studying English in college in China. With the introduction of AI and 5G, English classrooms are now intelligent and efficient for studying English. Gao [11] has offered research in the 5G era to find out how current technology may be applied to the English major at one of China's institutions. It is particularly advantageous in teaching English to assist students to access relevant information simply and without any limits, due to the faster transmission rate and various excellent web resources. The author in [12] presented a study to investigate the efficiency of mobile-assisted language learning in improving listening abilities for both teachers and students, as well as to determine the benefits of using MALL in language learning. To reduce the strain and raise the productivity of English teaching and learning, Zhu [13] has proposed research to construct and improve intelligence-based English classrooms. The teacher can set up video classrooms and use data technologies to assess the students using the proposed system's interface. Students can solve tasks and assess their learning levels to assess their abilities and knowledge. Hsu et al. [14] have developed a chatbot for English learners to practice speaking English through an online system called TPBOT. The findings indicate that it is a highly effective and productive method for learning oral English. The students who took part in the experiments improved their speech abilities significantly. Using artificial intelligence (AI) and 5G net technologies, this work develops a routing system called modernized energy-optimized LEACH protocol (M-LEACH). The system is capable of giving on-the-spot evaluation and constructive feedback. The VAE has been used to extract the features, and an RF classifier is used to accurately classify these features. Finally, the results are analyzed and compared to other approaches currently in use.

## 3. Proposed Work

This study introduces a modernized energy-optimized LEACH protocol using AI and 5G net technologies. A dataset of 6,600,000 items, containing 3,250,000 favorable and unfavorable texts in English was employed. The dataset is preprocessed using normalization to eliminate the impulse noises. Every single item in our assessment data set was gathered and analyzed from English website domains before being categorized as positive or unfavorable. Discriminant features are extracted using a VAE, and an RF classifier is used to classify the features with accurate performance. For better transmission of information, the M-LEACH routing algorithm is used in the 5G net service. Finally, the performances are examined, and the result is compared with other existing methods. The result is obtained using the MATLAB R2015 software.  Figure 1 depicts the framework of the proposed work.

### 3.1. Preprocessing

The data received is unfiltered, and it may contain a fake datagram as well as insufficient information. The data is cleaned and normalized to remove recurrent and redundant sounds, as well as insufficient data. Because the university community's records are so massive, specimen compaction techniques are used. Sine this dataset has several features, image retrieval methods are employed to sort out the ones which are not significant. The dataset is normalized during the preprocessing stage. Equation (1) defines the c-count in mathematical form as

(1) $$\begin{array}{c} C=\left[\frac{\left(M-\beta \;\right)}{\tau }\right], \end{array}$$

where *β* express the mean of the information, *τ* hints the standard deviation, and C is represented as

(2) $$\begin{array}{c} C=\frac{M-\bar{M}}{Sd}, \end{array}$$

where $\bar{M}$ points out the mean of the specimen, and Sd is the standard deviation of the specimens. The random specimen can be expressed as

(3) $$\begin{array}{c} C_{k}=\delta_{0}+\delta_{1}M_{r}+\rho_{r}. \end{array}$$

The defects that are depending on *τ*^2^ are represented by *r*.

Ensuring that, as seen below, the defects should not depend on one another.

(4) $$\begin{array}{c} t_{m}∼\sqrt{U}\frac{t}{\sqrt{t^{2}+u-1}}, \end{array}$$

where *t* implies the random parameter.

Next, the standard deviation is used to standardize the variable's moves. The momentary scale deviation is calculated using the following equation:

(5) $$\begin{array}{c} \text{MMS}=\frac{\mu^{\text{mms}}}{\theta^{\text{mms}}}. \end{array}$$

Here, the momentary scale is denoted by mms.

(6) μmms=ExM−β^MMS,

where *M* stands for a random variable, and Ex stands for expected values.

(7) θmms=ExM−β^MMS^2,tu=mmsM¯.

The coefficient of variance is denoted as *t*_*u*_.

The characteristic scaling procedure is stopped by setting all of the parameters to 0 or 1. The unison-based normalizing approach is employed which is computed as

(8) $$\begin{array}{c} M^{\prime }=\frac{\left(t-t_{\text{min}}\right)}{\left(t_{\text{max}}-t_{\text{min}}\right)}. \end{array}$$

The information can be kept after it has been normalized, and the length and irregularity of the information could be preserved. The normalized data are used as input in the subsequent steps.

### 3.2. Feature Extraction Using Variational Autoencoder

VAE is a deep Bayesian architecture that incorporates both neural network models and analytics [15, 16]. It also forces the underlying signals to pursue a specified allocation, like the Gaussian distribution, as opposed to the typical autoencoder. This change improves the learned aspects' ability to meet the demands of our target. The fundamental principle of VAE is introduced in this phase.  Figure 2 depicts the interior workings of VAE.

The encoder component of the neural network is supposed to show the conditional probability as

(9) $$\begin{array}{c} q_{w}=\left(u|o\right), \end{array}$$

where *o* represents the authentic information, *w* is the encoder's weight, and *u* shows the inherent codes.

Unlike other autoencoders, the VAE pushes the underlying codes *u* dispersion to resemble a conventional normal distribution. As an outcome, the underlying codes have persistent analytical features, making the decoder easier to use and our operation more efficient. The decoder then uses the underlying codes to try to obtain the model information. A neural network with weight, for example, *γ* indicates a conditional probability:

(10) $$\begin{array}{c} P_{\gamma }=\left(o|u\right). \end{array}$$

A new VAE technique is implemented. The decoder's sources are taken from the distribution of underlying codes to maintain ambiguity within the networks. The encoder is then programmed to produce two factors: the underlying codes' average and deviation vector. The two factors are then used to create a normal distribution to select a signal for the decoder. The entire layout of VAE is depicted in Figure 3.

### 3.3. Classification Using RF Classifier

In this section, a feature weighting method is presented for subdomain selection in random forests. We take an N-dimensional feature set {*B*_1_,  *B*_2_,…, *B*_*N*_}. For each feature in the field, we show how to calculate the weights {*U*_1_,  *U*_2_,…, *U*_*N*_}. These parameters are then utilized in a new method to create every random forest tree structure.

We assessed the source credibility of every incoming characteristic B as its relation to the class feature *Z* to calculate the characteristic weight. A high weight shows that item class labels in the training phase are associated with feature values *B*. As a result, *B* is useful for item class labels and has a high predictive opportunity for future item class labels. We suggest using chi-square techniques to calculate weight values to tackle multiclass issues. *B* is segmented using a smart linearization approach if *B* is quantitative. The chi-square statistical-dependent association is calculated using the table of characteristic B and the class characteristic *Z* of a set of data S as follows:

(11) $$\begin{array}{c} Cor\left(B,Z\right)=\sum_{m=1}^{e}\sum_{n=1}^{f}\frac{{\left(o_{mn}-w_{mn}\right)}^{2}}{w_{mn}}, \end{array}$$

where *o*_*mn*_ is the observed frequency, and *o*_*mn*_ represents the expected frequency.

The larger cor (*B*, *Z*) measurement, the more instructional characteristic B is regarding the class characteristic *Z*, and the greater the weight attributed to characteristic *B*.

Component weights are standardized for feature subdomain selection in practice. For *i* = 1,…, *K*, suppose the relationship between a characteristic *A*_i_ and the class label data *Y* is cor(*B*_*i*_, *Z*).

(12) $$\begin{array}{c} U_{i}=\frac{\sqrt{cor\left(B_{i},Z\right)}}{\sum_{i=1}^{K}\sqrt{cor\left(B_{i},Z\right)}}. \end{array}$$

Correction is commonly done by extracting the square root of the correlation. The normalized weight *U*_*i*_, as shown, determines the actual validity of characteristic *B*_*i*_. When constructing the proposed method, this weighted info is employed in the feature subdomain selection.

Next, the tree selection is performed. The most difficult aspect of the tree selection procedure is determining how accurate every tree is. To assess the relevance of a tree, we utilized out-of-bag reliability as a metric. The bagging technique is used to obtain a sequence of training data subgroups in a random forest process, and these training subgroups are subsequently utilized to construct trees. The training sample group used to develop the tree in each tree is referred to as an in-of-bag (IOB) sample, while the info group generated from the rest of the data is referred to as out-of-bag (OOB) info. Because OOB info is not utilized to create trees, it can be used to evaluate every tree's OOB correctness, and this OOB reliability can be used to determine the tree's relevance. The tree's OOB reliability, *t*_*l*_(IOB_*l*_), is defined as

(13) $$\begin{array}{c} {\text{OOBR}}_{l}=\frac{\sum_{i=1}^{k}\text{In}\left(t\left(s_{i}\right)=z_{i};s_{i}\in \;{\text{OOB}}_{l}\right)}{\sum_{i=1}^{k}\text{In}\left(s_{i}\in {\text{OOB}}_{l}\right)}. \end{array}$$

Here, indicating function is denoted by In(…). The greater the OOBR is the better the tree will be constructed. The trees are then sorted in descending order of their OOB precision, and the top 85% of trees are chosen to form the random forest. This type of tree choice can result in a community of “excellent” trees.

In this study, the proposed random forest method incorporates characteristic weights and tree selection techniques. Algorithm 1 introduces the framework of the proposed approach. The trained set of data, the feature set, the category characteristic, the number of trees in the random forest, and the size of subbands are all used as input data. The cycle for creating *D* decision trees is represented in stages 1 through 5. Stage 2 of the cycle uses the bootstrap method to select the trained information and build the in-of-bag information set for developing a tree classifier and the out-of-bag information set for evaluating the tree classifier on out-of-bag reliability. To generate a tree classifier, Stage 3 uses the recursive function generateTree (). The fourth stage calculates the tree classifier's out-of-bag reliability using the out-of-bag information set. Following the cycle, stage 6 sorted all created tree classifiers in descending order of the out-of-bag precision. Likewise, stage 7 chooses the highest 85% of trees with the highest out-of-bag reliability scores and blends the 80% tree classifiers into a random forest model. In practice, 85% is adequate to obtain satisfying performance.

Component generateTree function is started by making an advanced node. The halt conditions are then tested to determine whether to restore to the higher node or divide this node. Whether this node is divided, the feature weighting approach is used to choose *c* characteristics at arbitrary as a subspace for node division. Such characteristics are utilized as options for generating the optimum partitioning division for the node. The generateTree function is performed repeatedly for every subgroup of the division to construct a new node beneath the existing node. The parental node is returned when a leaf node is generated. This cyclical procedure is iterated till the complete tree is created.

### 3.4. Modernized Energy-Optimized LEACH Protocol (M-LEACH)

Originally, a hierarchal approach was used in wired broadband to save power, but it was later adopted in wireless sensors networks (WSNs) to obtain a longer lifespan and lower power consumption. The first adaptable protocol used in WSN for cluster head selection is M-LEACH. The M-LEACH is a round-based random dispersion, self-organize, and regular group identification approach [17, 18]. The major goal of the M-LEACH protocol is to reduce energy usage [19], which can be accomplished by carefully selecting groups in two stages: setup and steady state. M-LEACH separates the nodes into groups based on their random process. There will be a commanding head for each, which will be in charge of info transfer. The base station sends a report to all control nodes, or cluster heads (CHs), during the setup stage. As indicated in (14), these CHs are chosen based on the threshold value Th (m), which incorporates the likelihood of becoming CHs pr, the present round *r*, and the remaining of non-CHs in the previous 1/pr cycles.

(14) $$\begin{array}{c} \text{Th}\left(m\right)=\left\{\begin{array}{cc} \frac{pr}{1-pr\left(\text{ranmod}\left(1/pr\right)\right)}, & m\in g,\\ 0, & \text{otherwise}. \end{array}\right) \end{array}$$

The network randomly generates a value between all of the nodes as zeros and ones. If the produced value is less than Th(*m*), that node will serve as the cluster's control node, with the rest of the nodes serving as noncluster heads. The noncluster heads receive a request from the cluster head to connect the group for information transfer in phase 2 of steady state. The information is then sent from the CH to the sink node via non-CH channels. When choosing the CHs, although, node position and residual battery quantities are not taken into account. This routing algorithm is depicted in Figure 4.

## 4. Result and Performance Analysis

We have employed a MATLAB simulator in this study to examine and compare the behavior of the proposed protocol with the existing protocols. In this article, the main objective is to optimize the routing protocol for the better transformation of info. The performances such as the number of alive nodes and packets received, energy consumption, and transmission rate of the proposed protocol are examined and compared with other existing methods. These results are simulated in the MATLAB tool.

### 4.1. Transmission Rate

The transmission rate represents the number of bits per second. It is measured in megabits per second (Mbps). It also determines how long a signal stays on the transmission line.  Figure 5 depicts the transmission rate per every node of the M-LEACH protocol and provides a comparison of transmission rates for existing and proposed methods. When compared to other existing protocols, our proposed technique has a higher transmission rate. With an increase in the number of transmitting nodes, the transmission rate is significantly increased. This paper proves a higher transmission rate than the existing methods for each node to get higher data transmission.

### 4.2. Alive Nodes

The term alive node refers to a node that is always evolving. The term “dead node” refers to a node that can no longer be extended.  Figure 6 depicts the line of the number of alive nodes per round in the network. It is clear that with an increase in the number of rounds, there is only small degradation in the number of alive nodes. This shows that the proposed protocol can still provide high performance even if the number of rounds is increased.

### 4.3. Energy Consumption

The energy consumption of a base station is calculated by multiplying the effective return of the node's power usage by the duration of the event. In contrast to the broadcast and power bases, the energy required is the amount of energy consumed on data collection and evaluation. This is the amount of energy expended by the wireless transceiver.  Figure 7 provides the rate of energy consumption in Joules per round.

### 4.4. Network Packets

A network packet is a short piece of data that are transferred over a network using TCP. On the web or other packet-switched routes, a packet is the sequence of bytes transported between a source and a target.  Figure 8 depicts the number of received packets. It is evident that there is a linear trend between the number of packets received and the number of rounds. The number of the packet sent is significantly increased with an increase in the number of rounds. This shows that the proposed method can send more data as compared to other methods.

Figures 9–11 provide comparative results for power utilization, amount of received packets, and alive nodes with existing methods. We proved that the proposed method consumes minimum power as compared to other methods including the methods of RBM [16], NS2 [17], adjacent sensors [18], and LEACH-TM [19] as shown in Figure 9. When matched with existing methods, Figure 10 illustrates that the proposed method has a large amount of obtained network packets, and similarly, Figure 11 describes the less amount of expanded nodes in the proposed study as compared to the existing methods.

## 5. Conclusion

The application of AI-based systems and the 5G has carried out revolutions in education for both teachers and students. With the online learning platforms based on AI techniques, 5G has renovated the teaching and learning methods by charming and faster access to educational content. In this study, a routing protocol called modernized energy-optimized low-energy adaptive clustering hierarchical protocol was proposed using AI and 5G Internet technologies for online English teaching. The dataset was comprised of 6,600,000 items, including 3,250,000 favorable and unfavorable texts of the English language. The contents of the dataset were normalized to eliminate impulse noises, and a VAE was used to extract distinct features. For classification, an RF classifier was used to classify the features with accurate performance. The performance of the protocol was measured in terms of transmission rate, alive nodes, energy consumption, and the number of transmitted packets. Results show that the proposed M-Leach protocol provides a high transmission rate, more alive nodes, and minimum energy consumption as compared to other protocols. This study has provided a comprehensive picture of the prominent role of 5G and AI in English situational teaching in higher education for challenges of modern learning and the use of technology.

## Figures and Tables

**Figure 1:** Proposed work.

**Figure 2:** VAE interior workings.

**Figure 3:** The entire layout of VAE.

**Figure 4:** M-LEACH protocol algorithm.

**Figure 5:** Transmission rate.

**Figure 6:** Number of alive nodes.

**Figure 7:** Energy consumption (J).

**Figure 8:** Number of packets received.

**Figure 9:** Comparison of energy consumption J in suggested and existing methods.

**Figure 10:** Comparison of number of packets received in suggested and existing methods.

**Figure 11:** Comparison of number of alive nodes in suggested and existing methods.

**Algorithm 1:** Random forest classification algorithm

## Data Availability

The data used to support the findings of this study are included in the article.
